# A Chinese Medicine Compound Alleviates Cisplatin-Induced Acute Kidney Injury via Its Antiapoptosis and Anti-Inflammation Effects in Mice

**DOI:** 10.1155/2022/7841284

**Published:** 2022-06-29

**Authors:** Riming He, Jiahui Liu, Yulian Chen, Yijiao Liao, Yuzhi Wang, Xiaoming Jin, Zhongtang Li, Siqi Liu, Jiandong Lu, Shudong Yang

**Affiliations:** ^1^Department of Nephrology, Shenzhen Traditional Chinese Medicine Hospital, Guangzhou University of Chinese Medicine, Shenzhen, Guangdong, China; ^2^Shenzhen Traditional Chinese Medicine Hospital Affiliated to Nanjing University of Chinese Medicine, Shenzhen, Guangdong, China

## Abstract

Cisplatin, also known as cis-diamine dichloroplatinum (CDDP), is a widely used chemotherapeutic drug. However, its application is limited by the occurrence of serious nephrotoxicity. Currently, no effective therapy is available for combating CDDP-induced acute kidney injury (AKI). In the present study, we investigated the efficacy of Jianpi Yishen Tang (JPYST), a traditional Chinese medicine (TCM) compound commonly used to treat chronic kidney disease, against CDDP-induced AKI. In the CDDP + JPYST group, male mice were pretreated with JPYST (18.35 g/kg/day) for 5 consecutive days before receiving a single dose of CDDP (20 mg/kg), all mice were sacrificed 72 h after the CDDP injection. Results showed that JPYST suppressed CDDP-induced kidney dysfunction and tubular damage scores in the mice. Mechanistically, JPYST treatment attenuated CDDP-induced renal tubular cell apoptosis in AKI mice, as manifested by a marked decreased in TUNEL-positive cell counts, downregulation of the pro-apoptotic proteins Bax, Bad and caspase 3, and upregulation of the antiapoptotic protein Bcl-2 in kidney tissues. Meanwhile, JPYST decreased the expression of inflammatory cytokines TNF-*α*, IL-1*β*, and IL-6 in the serum and renal tissues of mice following CDDP administration. These factors are involved in suppressing the activation of phospho-NF-*κ*B p65 in tubular epithelial cells. Taken together, these findings demonstrated that JPYST exerts renoprotective effects against CDDP-induced AKI through antiapoptosis and anti-inflammation effects, and these are associated with downregulation of NF-*κ*B activation. Therefore, JPYST has potential for development of treatment therapies against CDDP-induced AKI.

## 1. Introduction

Cisplatin, also known as cis-diamine dichloroplatinum (CDDP), is a widely used chemotherapeutic drug for treating various solid tumors [1]. However, its application is limited by the occurrence of serious toxic side effects, the key among them being nephrotoxicity [2]. Previous studies have shown that approximately one-third of all patients administered with CDDP will suffer from renal injury due to the lack of effective prevention and treatment measures [3, 4]. CDDP-induced acute kidney injury (AKI) causes considerable mortalities and morbidities globally [5]. The existing regimens, such as aggressive hydration and forced diuresis for the treatment of CDDP patients do not completely prevent the development of CDDP-induced AKI [6], necessitating urgent development of efficacious and safe therapies.

Numerous studies have shown that apoptosis and renal inflammation play an important role in pathological process of CDDP-induced AKI [7, 8]. Particularly, excessive apoptosis of tubular epithelial cells (TECs) has been implicated in tubular necrosis and renal dysfunction. In the intrinsic (mitochondrial) apoptotic pathway, tubular CDDP accumulation causes activation of BCL2 apoptosis regulator family proteins, thereby inducing AKI [9, 10]. Moreover, inflammation is closely correlated to the progression of CDDP-induced AKI, with recent studies revealing that inhibition of inflammatory mediators can effectively attenuates CDDP-induced AKI [11]. The transcription factor nuclear factor-*κ*B (NF-*κ*B) has been considered a key regulator of inflammation and apoptosis in CDDP-induced AKI [12]. In this context, antiapoptotic and anti-inflammatory agents have become primary approaches to combat CDDP-induced nephrotoxicity. Recently, formulations of traditional Chinese medicine (TCM) compounds have exhibited potential protective effects against CDDP-induced renal damage [13–15].

In particular, Jianpi Yishen Tang (JPYST) is a traditional Chinese medicine compound commonly used to treat chronic kidney diseases along with its complications [16–21]. In our previous studies, it was observed that JPYST protects 5/6 nephrectomized rat kidney from damage via suppression of inflammatory responses by inhibiting the NF-*κ*B activation and mediating downregulation of proinflammatory mediators *in vitro* [20, 21]. To date, however, efficacy as well as the underlying mechanisms of JPYST on treatment of CDDP-induced AKI remain unclear. The present research aimed to evaluate the efficacy of JPYST on suppressing CDDP-induced AKI and elucidate the underlying mechanisms of action. Our results demonstrated that JPYST exerts an antiapoptotic potency and has a protective function against CDDP-induced AKI.

## 2. Materials and Methods

### 2.1. Preparation of JPYST

JPYST was prepared according to a previously described method as in Reference [20]. Briefly, eight herbs of JPYST were weighed, then extracted twice in 1200 ml of boiling water for 60 minutes. The contents were centrifuged, the supernatant was collected, and then decompressed and dried. The resulting powder was stored at −80°C. The JPYST power was redissolved in ultrapure water under room temperature prior to administration.

### 2.2. Animals and Experimental Treatment

All animal experimental and feeding protocols were approved by the Animal Ethics Committee of Guangzhou University of Chinese Medicine. Male C57BL/6J mice, 8 weeks old, and weighting between 20–25 g, were purchased from Nanjing Biomedical Research Institute of Nanjing University. The animals were maintained under a controlled room at temperature, with air conditioning and a 12 h light//12 h dark regime. They were also allowed free access to food and drinking water. One week after the acclimatization, 15 mice were separated into 3 groups, namely, the control group (*n* = 5), CDDP (*n* = 5), and CDDP + JPYST (*n* = 5) groups. Mice in the CDDP and CDDP + JPYST groups were administered with a single dose of 20 mg/kg CDDP (Sigma-Aldrich, USA) via intraperitoneal injection, while those in the control group received an equal volume of distilled water. Those in the AKI + JPYST group were pretreated with JPYST (18.35 g/kg/day) via intragastric gavage for 5 consecutive days before CDDP injection. All mice were sacrificed 72 h after the CDDP injection and their blood and kidneys were harvested for biochemical and histopathological analysis (Figure 1(a)).

### 2.3. Analysis of Serum Parameters

Serum creatinine (Scr) and blood urea nitrogen (BUN) were measured by the Scr detection kit and BUN detection kit (StressMarq Biosciences, Canada), respectively, according to the manufacturer's instructions.

### 2.4. Histological Analysis

Mice were sacrificed, their renal tissues were collected, fixed in 10% buffered formalin, and embedded in paraffin. Sections (3 *μ*m-thick) were sequentially stained in periodic acid Schiff (PAS) followed by the evaluation of kidney's pathological damage under a light microscope. Tubular damage in PAS staining sections was scored as follows: 0 = normal; <10% damage = 1; 10%–25% damage = 2; 26%–75% damage = 3; and >75% damage = 4. Tubular damage was defined as a loss of brush border, blistering of the apical membrane, or accumulation of cells and proteins in the lumen.

### 2.5. Western Blot Analysis

Proteins from renal tissues were extracted using the RIPA lysis buffer (Thermo Fisher, USA) and quantified using the BCA Protein Assay Kit (Thermo Scientific, USA). Equal concentrations of proteins were separated on 10 or 15% SDS-polyacrylamide gels and were subsequently transferred to a PVDF membrane (Millipore, USA). The membranes were blocked using 5% nonfat milk for 60 min, under room temperature, then incubated overnight with primary antibodies at 4°C. In order to bind primary antibodies, HRP-conjugated secondary antibodies were incubated for 60 min under room temperature. Blots were detected and visualized with Clarity Western ECL Substrate (Bio‐Rad) under a MP imager (Bio‐Rad developed). Density analysis of the protein bands was performed using Image Lab 5.1 which was used for (Bio-Rad, USA). The primary antibodies used in the study were against the proteins and included the following: rabbit anti-cleaved caspase-3 (1 : 250) (Cell Signaling Technology, USA), rabbit Anti-Bad (1 : 1000), rabbit Anti-Bax (1 : 1000) (Abcam, USA), rabbit Anti-GAPDH (1 : 1000) (Cell Signaling Technology, USA), rabbit Anti-p-p65(Ser536) (1 : 1000) (Cell Signaling Technology, USA), and mouse anti-*β*-actin (1 : 5000) (Sigma-Aldrich, USA).

### 2.6. Measurement of Inflammatory Cytokines

The mouse plasma was centrifuged and the supernatant was used to determine the level of inflammatory cytokines. The concentrations of TNF-*α*, IL-6, and IL1-*β* were measured by a Milliplex MAP Mouse Cytokine/Chemokine Panel (Millipore Corporation, MA, USA) on the Luminex-200 platform. Data analysis was performed with Milliplex Analyst 5.1 software (Millipore Corporation, MA, USA) [20].

### 2.7. Quantitative Real-Time PCR (qRT-PCR)

Mouse renal tissues were collected and total RNA was extracted using the RNA Easy Fast Tissue/Cell Kit (TianGen, Beijing, China) according to the manufacturer's instructions. RNA was reverse-transcribed into cDNA using the PrimeScript™ RT Master Mix (Takara, Japan) according to the manufacturer protocol. The mRNA level of TNF-*α*, IL-1*β*, IL-6, and GAPDH were assessed using the SYBR® Select Master Mix (Applied Biosystems, USA) and ABI QuantStudio 5 Real-Time PCR System (Applied Biosystems, USA) according to the manufacturer's instructions. The relative gene expression level was quantified using the 2^−ΔΔCt^ method and the expression was normalized to that of GAPDH. The sequences of the gene-specific primers (TsingKe Biotechnology, Beijing, China) used in this study are shown in Table 1.

### 2.8. Immunohistochemical Staining (IHC)

Deparaffinized and hydrated sections (3 *μ*m thick) were first pretreated with sodium citrate buffer (0.01 M, pH 6.0) in a water bath (95°C, 30 min) for unmasking of antigens, and then exposed to 3% hydrogen peroxide for 20 min to quench endogenous peroxidase activity. Thereafter, they were incubated in 10% goat serum for 30 min under room temperature, followed by overnight incubation with primary antibodies, including Bcl-2(1 : 200), p-p65 (Ser536) (1 : 50), and p65 (1 : 50) (Cell Signaling Technology, USA) at 4°C. Subsequently, the sections were washed and incubated with a SignalStain Boost IHC Detection Reagent (Cell Signaling Technology, USA) for 1 h, then, SignalStain diaminobenzidine (DAB) substrate (Cell Signaling Technology, USA) was added to develop a brown color. The sections were photographed under an optical microscope (Carl Zeiss, Germany). Three kidney specimens from each group were blindly captured across four equal microscopic fields (400x). For quantitative analysis, we performed integrated optical density (IOD) measurements on immunohistochemistry images to calculate average optical density (AOD) using the equation AOD = IOD/area. After defining the region of interest, the AOD of the selected area (IOD per unit area) was determined using Image-Pro Plus 6.0 software. The AOD represents the protein immunoreactivity within the renal tissue.

### 2.9. Terminal Deoxynucleotidyl Transferase dUTP Nick End-Labeling (TUNEL) Assay

Cellularapoptosis in renal tissues was detected using TUNEL staining according to the manufacturer's instructions (Beyotime Biotechnology, China). Briefly, 4 *μ*m-thick paraffin embedded kidney sections were dewaxed and rehydrated. Then, the sections were incubated with proteinase K (Beyotime Biotechnology, China) at room temperature and rinsed with PBS. After treatment with 3% H2O2 for 20 min at room temperature, the sections were incubated with a TUNEL reaction mixture for 1 h at 37°C in the dark. Subsequently, slides were developed with 3,3′-diaminobenzidine (DAB; Beyotime Biotechnology, China) for 3 min and nuclei were counterstained with hematoxylin (Solarbio, China). For quantification, TUNEL-positive cells were counted in 6 non-overlapping 400x microscopic fields from each animal per group.

### 2.10. Statistical Analysis

Statistical analyses were performed using GraphPad Prism 8.3.0 and data are represented as means ± standard errors of the mean (SEM) from at least 3 independent experiments. Differences among groups were evaluated using one-way analysis of variance (ANOVA) followed by Tukey's post hoc test for mean separation. Statistical significance was set at *P* < 0.05.

## 3. Results

### 3.1. JPYST Suppresses the CDDP-Induced Renal Dysfunction and Histopathological Damage

To analyze the effects of JPYST on progressive of acute kidney injury (AKI), we established a cis-diamine dichloroplatinum (CDDP)-induced AKI mouse model. Results from periodic acid-Schiff (PAS) staining revealed a significant increase tubule injury score in CDDP-treated mice compared to those in the control group. On the other hand, histological features of the injury included tubular cell swelling and sloughing, loss of brush border, tubular dilation, as well as cast formation. Moreover, JPYST markedly improved these pathological changes (Figures 1(b) and 1(c)). Notably, the blood urea nitrogen (BUN) levels were significantly higher in the CDDP group (17.36 ± 0.59 mg/dl) than those of the controls (2.43 ± 0.11 mg/dl, *P* < 0.0001), which was consistent with the tubule injury scores. In addition, we observed significantly higher serum creatinine (Scr) levels in mice in the CDDP group (3.42 ± 0.35 mg/dl) than those in the control (1.07 ± 0.06 mg/dl, *P* < 0.0001). Strikingly, the administration of JPYST significantly attenuated the increase in BUN and Scr levels (*P* < 0.0001) (Figures 1(d) and 1(e)).

### 3.2. JPYST Ameliorates the CDDP-Induced Renal Apoptosis Level

Numerous evidence has demonstrated that tubular epithelial cell apoptosis is an important feature of AKI induced by nephrotoxic drugs [9, 10]. Therefore, we analyzed a range of apoptosis-associated proteins to elucidate the renoprotective role of JPYST on CDDP-induced apoptosis in renal tissues of mice. The TUNEL assay revealed a significant increase in TUNEL-positive cell count in renal of CDDP treatment grounds mice as compared to that of the control ground mice; the TUNEL-positive cells were distributed primarily in the renal cortex, especially in the renal tubules. Treatment with JPYST greatly reduced the count of TUNEL-positive cells (Figures 2(a) and 2(b)). Moreover, Western blot analysis and IHC staining demonstrated a markedly upregulation of cleaved-caspase-3 protein (which plays a key role in the executive stage of apoptosis) as well as Bax and Bad proteins (critical regulators of apoptosis-associated proteins), while downregulating the anti-apoptotic protein BCL-2 in the CDDP group relative to controls; Bcl-2 was mainly expressed in the cytoplasm of renal tubular epithelial cells (Figures 2(c)–2(h)). Interestingly, the administration of JPYST for 5 consecutive days before being sacrificed effectively reversed these changes.

### 3.3. JPYST Inhibits the Expression of Inflammatory Cytokines

Previous studies have shown that inflammation is closely associated with the progression of CDDP-induced AKI [11]. Based on this, we examined whether JPYST downregulates proinflammatory mediators in serum and renal tissues. Serum levels of cytokines TNF-*α*, IL-1*β*, and IL-6 were upregulated by cisplatin but were markedly reduced by JPYST (Figures 3(a)–3(c)). In agreement with the results obtained with serum cytokines, qPCR data also indicated that the mRNA expression of TNF-*α*, IL-1*β*, and IL-6 were greatly induced by cisplatin, which was significantly decreased after JPYST treatment (Figures 3(d)–3(f)). These results demonstrate that JPYST inhibited the expression of inflammatory cytokines in the serum and renal tissues of CDDP-induced AKI mice.

### 3.4. JPYST Suppresses NF-*κ*B Activity

NF-*κ*B is considered a key regulator of inflammation and apoptosis [12]. To further elucidate the molecular mechanism underlying the anti-inflammatory and antiapoptotic effects of JPYST, we next examined that its treatment could suppress the NF-*κ*B signaling pathway, by measuring levels of NF-*κ*B p65 (p65) and phospho-NF-*κ*B p65 (p–p65). Results from immunohistochemical analyses of kidney sections revealed a significantly increased expression of p65 and p–p65 in the CDDP group relative to controls; p65 and p–p65 positive staining predominately localize to renal cortex tissues, especially in the cytoplasm of damaged tubular epithelial cells; Western blot analysis showed a significantly upregulation of p–p65 protein in the CDDP group. Interestingly, the activity of p65 and p–p65 in the mice treated with CDDP + JPYST was significantly diminished (Figure 4), indicating that the JPYST exerts its anti-inflammatory and antiapoptotic effects by regulating the NF-*κ*B signaling pathway in the CDDP-induced AKI mice.

## 4. Discussion

In the present study, we have illustrated that Jianpi Yishen Tang reversed renal dysfunction and reduced renal tubular cell apoptosis and inflammation in CDDP- induced AKI in a mice model. These renal protective effects of JPYST on CDDP-induced AKI may be mediated through antiapoptosis and anti-inflammation mechanisms and are associated with the activation of the NF-*κ*B signaling pathway. AKI, whose occurrence is accompanied by a high rate of morbidity and mortality due to lack of effective prevention and treatment therapies, is a serious complication of CDDP therapy [3]. Therefore, there is a need to urgently develop effective approaches for prevention and control measures. To date, however, no effective therapy is available for combating CDDP-induced AKI.

JPYST is a traditional Chinese medicine with strong biological and pharmacological activities. Results from our previous studies showed that JPYST protects 5/6 nephrectomized rat kidneys from damage by suppressing inflammatory responses through the inhibition of NF-*κ*B activation, as well as mediating downregulation of proinflammatory mediators *in vitro* [20, 21]. However, the underlying mechanisms of JPYST's action on CDDP-induced AKI remain unclear.

Numerous studies have demonstrated that excessive apoptosis and inflammation are among the underlying mechanisms for development of CDDP-induced AKI. In fact, antiapoptosis and anti-inflammation of kidney tissues were confirmed to exert protective effects on CDDP nephrotoxicity [7, 8]. Specifically, excessive TECs apoptosis contributes to tubular necrosis and renal dysfunction. On the other hand, Bad and Bax, important members of the Bcl-2 family are key regulators of mitochondrial permeability and caspase-3 activation. In the internal (mitochondrial) apoptotic pathway, the TEC injury mediates activation of proapoptotic Bad and Bax proteins, thereby inducing AKI [22, 23]. Results of the present study revealed that antiapoptotic Bcl-2 expression markedly decreased, while proapoptotic Bad, Bax, and caspase-3 expression increased in CDDP-treated AKI mice. Interestingly, JPYST treatment attenuated CDDP-induced renal tubular cell apoptosis in AKI mice, as manifested by a marked decrease in TUNEL-positive cell counts, downregulation of the Bax, Bad, and caspase 3, and upregulation of protein Bcl-2 in kidney tissues. These results indicate that JPYST exerts renoprotective effects by inhibiting CDDP-induced renal cell apoptosis.

Previous studies have shown that renal tissue inflammation is a crucial feature in the pathogenesis of CDDP-induced AKI [11, 24, 25]. For example, CDDP accumulation in tubular cells was shown to promote the recruitment and infiltration of inflammatory cells in renal tissues, thereby upregulating proinflammatory mediators such as TNF-*α*, IL-6, and IL1-*β*. These findings affirm its involvement in AKI progression [26, 27]. Our results revealed significant upregulation of TNF-*α*, IL-6, and IL1-*β* in the serum and renal tissues of mice following CDDP treatment. In contrast, JPYST reversed this trend in the kidneys after CDDP administration. Overall, these results indicated that inhibiting production of inflammatory cytokines may be another mechanism through which JPYST improves CDDP-induced AKI.

NF-*κ*B is considered a key regulator of inflammation and apoptosis. CDDP increased the phosphorylation of NF-*κ*B in TECs, and these phosphorylated proteins increase the transcription of different proapoptotic and proinflammatory transcription factors, thus mediating an increase apoptosis and inflammation and causing kidney damage [28–31]. Results of the present study showed that JPYST inhibits the NF-*κ*B activation in TECs, indicating JPYST experts antiapoptotic and anti-inflammatory effects by suppressing the NF-*κ*B signaling pathway in CDDP-induced AKI.

In conclusion, JPYST can alleviate CDDP-induced AKI via its antiapoptotic and anti-inflammatory effects. Notably, these effects are associated with the suppression of NF-*κ*B activation in TECs, suggesting that JPYST could be a potential therapeutic agent for treatment of CDDP-induced AKI.

## Figures and Tables

**Figure 1:** JPYST suppresses CDDP-induced kidney dysfunction and histopathological damage. (a) Diagram of the experimental protocol. (b) and (c) Representative kidney sections stained with periodic acid-Schiff and quantitative analysis of renal tubular injury in different groups of mice. Scale bar, 50 *μ*m (overview) and 20 *μ*m (inset). (d) and (e) Levels of serum BUN and creatinine across different groups of mice. Data presented are means ± SEM (*n* = 5). ^*∗∗∗*^*P* < 0.001, ^*∗∗∗∗*^*P* < 0.0001.

**Figure 2:** JPYST ameliorates CDDP-induced renal apoptosis levels. (a) Apoptosis of renal tissue sections was analyzed by the TUNEL assay. Arrows show TUNEL-positive cells in renal tubular area (400x). Scale bar, 100 *μ*m. (b) Quantification of TUNEL-positive cells in cortical renal tubular. (c) Western blots showing patterns of cleaved-caspase-3, Bad, and Bax protein expressions in renal tissues. (d)–(f) Quantitative analysis of cleaved-caspase-3, Bad, and Bax protein expression in the renal tissues. (g) Representative immunohistochemistry (IHC) images of Bcl-2 protein in renal cortical glomeruli and tubular epithelium (400x). Scale bar, 100 *μ*m (h) Quantitative analysis of IHC for the Bcl-2 protein expression. AOD = IOD/area. Data presented are means ± SEM (*n* = 5).  ^*∗∗*^*P* < 0.01,  ^*∗∗∗*^*P* < 0.001,  ^*∗∗∗*^*P* < 0.0001.

**Figure 3:** JPYST inhibits inflammatory cytokine expression in CDDP-induced AKI mice. (a)–(c) Representative serum levels of cytokines TNF-*α*, IL-1*β*, and IL-6 in mice. (d)–(f) mRNA expression levels of TNF-*α*, IL-1*β*, and IL-6 in renal tissues were measured by quantitative real-time PCR. Data presented are means ± SEM (*n* = 5).  ^*∗*^*P* < 0.05,  ^*∗∗*^*P* < 0.01,  ^*∗∗∗*^*P* < 0.001,  ^*∗∗∗∗*^*P* < 0.0001.

**Figure 4:** JPYST suppresses NF-*κ*B activity in CDDP-induced AKI mice. (a) Representative IHC images of p65 and p–p65 in cortical renal tubular epithelial cells (400x). Scale bar, 100 *μ*m. (b), (c) Quantification of IHC for p65 and p-p65. AOD = IOD/area. (d) Western blots showing patterns of p–p65 protein expressions in renal tissues. (e) Quantitative analysis of p–p65 protein expression in the renal tissues. Data presented are means ± SEM (*n* = 5).  ^*∗∗*^*P* < 0.01,  ^*∗∗∗∗*^*P* < 0.0001.

**Table 1:** Gene-specific primers for qRT-PCR.

Gene name	Forward	Reverse
GAPDH	GGCAAATTCAACGGCACAGT	CGCTCCTGGAAGATGGTGAT
TNF-*α*	GGTGCCTATGTCTCAGCCTCTT	GCCATAGAACTGATGAGAGGGAG
IL-6 IL-1*β*	TACCACTTCACAAGTCGGAGGC TGGACCTTCCAGGATGAGGACA	CTGCAAGTGCATCATCGTTGTTC GTTCATCTCGGAGCCTGTAGTG

GAPDH, glyceraldehyde-3-phosphate dehydrogenase; TNF-*α*, tumor necrosis factor-*α*; IL-6, interleukin-6; IL-1*β*, interleukin-1*β*.

## Data Availability

The data used to support the findings of this study are available from the corresponding author upon request.
